RETRACTED

# Climate change and sustainable agricultural growth in the sahel region: Mitigating or resilient policy response?

**DOI:** 10.1016/j.heliyon.2023.e19839

**Published:** 2023-09-08

**Authors:** Ting Wang, Chengwu Sun, Zheqi Yang

**Affiliations:** a Faculty of Marxism, Northeast Normal University, Changchun, 130000, Jilin, China; b Hulunbuir Maritime Safety Bureau, Hulunbuir, 021000, Inner Mongolia, China

**Keywords:** Climate change, Greenhouse gas, Rainfall, Sustainability, Agriculture, Sahel region

## Abstract

The aim of this study is to provide an empirical answer to the question of whether nexus exists between climate change and sustainable agricultural growth in nine (9) countries within the Sahel region between 1990 and 2020. The study utilized Panel ARDL and Pairwise Dumitrescu Hurlin Panel Causality Tests to arrive at the following conclusions; firstly, the climate change orchestrated by change in rainfall is a very prominent factor causing reduction in sustainable agricultural growth in the Sahel region. One way feedback relationship flows from sustainable agricultural growth to greenhouse gas emission. In the light of the above, this study recommends that, in addressing the adverse effects of change in rainfall on agricultural sustainability, the policymakers in the Sahel region in particular and Africa as a whole should embark on a policy mix by embanking on mitigating policy response towards ensuring sustainable agricultural production via irrigation which is the best mode of water provisions without causing negative spilliovers on the environment. Also, the policymakers should be proactive by embarking on policies and programs that would build the resilience and adaptation of the region ahead of the future adverse effects of agriculturally induced climatic change.

## 1 Introduction

Over the past decades, the issues surrounding the aftermath effects of climate change on both humans and environment have become the major issue of concern among international policy agenda and public discussion [1]. These issues became more intense at the United Nations COP15 Conference in Copenhagen, December 2009. In the recent times, one of the critical submissions of the ﬁfth assessment report of the United Nations’ Intergovernmental Panel on Climate Change (IPCC) is the disastrous impacts of climate change on industries such as agriculture [2,3]. Change in climate has the tendency to cause disequilibrium in food supply which aggravating the challenge to meet ever increasing demand for food due to population explosion in the developing countries and continuous urban development in developed economies.

Consequently, climate change and its spillovers on sustainable agriculture have become the priorities of both the researchers and policymakers in countries in the Sahel region. Against this backdrop, an empirical insight of the nexus between climate change and sustainable agricultural growth was carried out.

RETRACTED

This study is very germane in the Sahel region because this sub region of Africa is in a dire state of vulnerability to the influence of climate change as a result of over reliance on a combination of biophysical factors and natural resources especially agriculture for economic survival of teeming population in this region. In the same vein, the structure of agricultural sector in the Sahel region is extremely underdeveloped [4], coupled with the recent continuous shortage of water resources fueling the persistent conflict among farmers, fishermen and herders in one hand, and high levels of insecurity of food, properties and lives in Burkina Faso, Chad, Niger, Mauritania, Mali and Nigeria [[5], [6], [7]].

It is imperative to argue that this study is novel in the sense that a policy driven empirical research focusing on climate change and sustainable agricultural growth within a panel analysis of countries in Sahel region is missing in the literature, to the best of our knowledge. However, several past studies revolving around climate change and its influence on agriculture such as Ayinde et al. [8] focusing on Nigeria. Other studies with coverage of Sahel region such as Busby [9] focusing on climate and security, Biasutti [10] focusing on trends of rainfall and Cooper [11] which only identifies opportunities that climate change adaptation and mitigation could drive. Hence, there is a huge existing gap in the literature for this study to fill.

Moreover, this current study is unique by providing empirical answer to the question what is the linkage between climatic parameter and sustainable agricultural growth within Sahel region. The justification for this study is that it would provide an empirically informed policy that would drive climate mitigation and adaptation vis-à-vis sustainable agricultural growth in the Sahel region. As such, this study is divided into these sections; introduction identifies the problem of the study and justifies it accordingly. Literature review provides detailed information about the past empirical studies as regard to the subject matter of this study. Whereas, the latter part of the paper discusses the methodology, results and the policy implications of the paper respectively.

## 2 Literature review

Using the Autoregressive Distributed Lag (ARDL) for the years 1982–2014, Chandio et al. [12] examined the short-term effects of climate change on agriculture in China. The findings demonstrated that temperature and rainfall have an unpleasant influence on agricultural product over the long term, CO2 emissions had a substantial impact on agricultural output in both immediate- and long-term assessments. The quantity of land devoted to cereal crops, the amount of fertilizer used, and the amount of energy consumed, among other factors, all significantly and positively influence agricultural production in both the long- and short-term.

RETRACTED

The impact of climate change on Nigerian agriculture and rural life was examined by Agbola and Fayiga [13]. According to the report, farmers may become discouraged and shift their livelihoods, particularly in rural areas, as a result of the fall in agricultural production. It was also discovered that agriculture might cause rural to urban migration, which would have an impact on the growth of the nation's rural districts.

In eleven (11) Southern and Eastern African (ESA) nations between 1961 and 2011, Belloumi [14] examined the effects of climatic change on agricultural contribution. The study indicated that while the general increase in annual mean temperature diminishes agricultural productivity in ESA, variable precipitation has a beneficial impact on agricultural output. The optimal adaptation and mitigation strategies may be chosen by policy makers with the aid of a quantified assessment of the effects of change of climate on agricultural productivity.

The difficulties of agricultural climate change adaptation in Nigeria were highlighted by Enete al [15]. The findings showed that rural Nigerians, who provide more than 70% of the country's food supply, are disproportionately impoverished and frequently suffer from hunger and illness. The government's initiatives to combat poverty, combat HIV/AIDS, and advance agricultural knowledge should not only be decentralized but also participative, according to the advice given.

Molua et al. [16] studied the influences of change in climate on African agriculture. The results imply that the four nations' agricultural returns are impacted by the climate. The findings also demonstrate a non-linear link between precipitation and agricultural revenue and between temperature and crop revenue. Overall, the temperature elasticity indicates that all countries' agricultural sectors are negatively impacted by global warming. An empirical examination of the impacts of global warming on farming activities of the Nigerian, and an assessment of the factors that propel adaptation to change of change are provided by Apata [17]. Primary sources alongside secondary sources provided the information used in this investigation.

Examining the coverage of the three scenarios was made possible by the collection of secondary data sources (1971–1980; 1981–1990 and 1991–2000). Only 850 of the 900 respondents in the initial data set were useable. In order to assess the consequences of fast climatic change on the cultivation of grain and the population of humans in Nigeria, this study examined the drivers of farm-level climate adaptation strategies using a multinomial choice and stochastic simulation model. According to the findings by Apata [17], if grain availability does not keep up with population expansion in an adverse climatic climate, hunger-related mortality may rise. The productivity of farms is, nevertheless, significantly impacted by climate change responses.

RETRACTED

The economic impacts of climate change on Southeast Asian nations until 2080 were evaluated by Zhai [18]. The findings imply that the overall effects of agricultural losses brought on by change of climate on the world economy are quite minor. The poor world would ultimately end up as a net loser as a result of the unequal distribution of productivity losses across global areas, which would lead to large structural modifications in global agricultural output and trade. A decline in agricultural productivity would have minor but not insignificant negative effects on Southeast Asia's economic production given the predicted decline in the agricultural sector of the economy.

Agricultural import dependency is predicted to rise in the next decades, the majority of Southeast Asian economies will see worsening terms of trade and greater welfare losses. The negative consequences are anticipated to vary by economic structure, being less severe for Malaysia as well as Singapore and more severe for, Indonesia, Viet Nam, Thailand and the Philippines. The region should focus on reverting its current pattern of diminishing agricultural output if it is to be able to manage the possible agricultural damages caused by the anticipated changes in climate.

Given the influence of change of climate on shifting livelihood patterns in the nation, Ayinde [19]. The study on the impact of change of climate on agricultural production is crucial. The time series data utilized in this paper were analyzed using descriptive and co-integration analytic methods. The results showed that between 1981 and 1995, the rate of agricultural production increase was consistently higher, followed by a substantially lower growth rate in the subperiod between 1996 and 2000. The trend in the pattern of rainfall varied. Also not consistently stable was the temperature. However, rains from the previous year had a substantial detrimental impact on this year's agricultural yield. It is advised that ecologically and agriculturally sensitive technology and developments that can minimize climatic fluctuation be supported if agricultural production was to be enhanced and sustained.

RETRACTED

Climate change and agricultural productivity in Nigeria were examined by Ayinde et al. [8] exploring time series data. The analytical techniques employed were granger causality test analysis and descriptive statistics. From 1987 through 2000, productivity was seen to be steadily increasing until declining in 2001. The growth may be attributed to a number of government initiatives and projects, including the Agricultural Development Program and the Lower Niger River Basin Development Authority (LNRBDA) (ADP). Whereas, the temperature is fairly stable and has little impact on the productivity of agriculture. Changes in rainfall (a climatic parameter) have a beneficial impact on agricultural productivity in Nigeria, according to the Granger causality theory. So it is advised that irrigation is the most appropriate method of water availability in order to boost and sustain agricultural productivity while minimizing environmental impact.

Using an integrated approach that includes environmental and socio-economic drivers during the period of 1951–2010, Atedhor [20] investigated the agricultural susceptibility to change of climate in eight chosen rural communities in Sokoto State of Nigeria. To investigate the association between the factors and the sampled farmers' agricultural vulnerability, multiple linear regression was performed. The problem of multi-collinearity in the independent variables was solved using stepwise regression, which further strengthened the model.

The findings by Atedhor [20] indicated that, despite decreased trends in Sokoto's annual rainfall and number of rainy days, annual mean temperatures are rising. During the time period under consideration, yearly droughts had mild to moderate intensity. The findings also revealed that eighty-six (86%) of the variance in agricultural susceptibility to climate change in the chosen communities in Sokoto State was caused by inconsistent rainfall, desertification, rising temperatures, a lack of pastures, and difficulty accessing credit facilities. Therefore, the article suggests that irrigation projects be developed, managed grazing be implemented, and sustainable local farmers be provided with soft and accessible lending facilities.

Onyeneke et al. [21] evaluated the sustainability and resilience of farmer-adopted solutions to mitigate the threats presented by climate change. 95 studies from the years 2010–2019 that focused on smallholder rural farmers' adaptation to climate change in Nigeria were systematically reviewed. Using the Ifejika-Speranza Resilience Check Toolkit, the study by Onyeneke et al. [21] evaluated the climatic resilience of the adaptation measures. The findings demonstrated that farmers are utilizing climate-resilient adaptation strategies; however, because the current study is not focused on sustainable agricultural systems, we were unable to determine how these strategies have resulted in them. Also, the results reveal that the bulk of adaptation studies in Nigeria are concentrated on the subsystem of crop farming. Crop farming, animal farming, and fish farming are the three main agricultural ecosystems and the three main adaption regions.

RETRACTED

The plan for agricultural adaptation to change of climate in Southern Nigeria was evaluated by Ozor [22]. The study was done in Southern Nigeria between 2008 and 2011 and had 360 respondents who were chosen using a multi-stage random sample approach. The majority of respondents (84%) knew that there had been an increase in land degradation as well as, pests, weed infestation and diseases. Other characteristics of change of climate included uncertainty at the start of the growing season, along side pests and diseases, then extreme weather scenarios like droughts and flooding. Declining soil fertility and plant infestation were the two most major consequences of climate change to be seen in the area.

By generating fixed effects models, Belloumi [23] examined the impact of climatic variables such as temperature precipitation on security of food 10 economies within Eastern and Southern Africa between 1961 and 2011. The findings demonstrate the importance of land used for grain production, population growth, inflation, and GDP per capita in explaining the indices of food security. While temperature has a detrimental impact on food security when it comes to climatic factors, total rainfall has a favorable and considerable impact. To lessen the effects of and adapt to climate change, policymakers will need to base their choices on the adoption of contemporary agricultural practices that maximize water utilization through expanded and enhanced irrigation systems and crop development.

Alboghdady and El-Hendawy [24] analyze the effects of climate change and variability on agricultural production in the Middle East and North Africa region by first conducting a Fixed Effect Regression (FER) analysis and then conducting a marginal impact analysis to determine the effects of these factors on agricultural production for the years 1961–2009. According to the findings, agricultural productivity decreased by 1.12% owing to a 1% rise of wintertime temperature. A further finding showed that a 1% increase in seasonal temperature variation throughout the winter and spring led to a 0.09 and 0.14% drop in agricultural output, respectively. The findings also showed that rising precipitation during the winter and fall seasons and precipitation unpredictability throughout the winter and summer seasons had a detrimental influence. According to the estimated squares of temperature and precipitation, the MENA region's agricultural contribution was largely propelled by change of climate in a nonlinear manner.

RETRACTED

The impact of climate change on Africa's food security was recently demonstrated by Pickson, and Boateng [25]. In order to examine patterns related to climate change, we used the Mann-Kendall test and Sen's slope estimator. In order to examine how change of climate has affected security of food in 15 African nations between 1970 and 2016, the researcher applied the pooled mean group approach and the Dumitrescu-Hurlin panel causality test. Three things were found through empirical research. First, a thorough examination shows that rainfall has a significant impact on Africa's food security. But across the 15 nations, there were significant differences in the importance of the impact of rainfall. Second, we discover that temperature has no significant long-term effect on security of food. The short-term outcomes, however, demonstrated that, albeit to various degrees across nations, severe temperatures pose a threat to food security.

By combining cross-sectional data gathered via a set of questionnaire in the Rawalpindi division together with time series data of meteorological variables acquired from metrological stations, the study by Shakoor [26] was able to track the effects of change of climate on the agriculture of dry regions. To examine the connections between Net Farm Revenue (NFR) and climate in the dry region, a Ricardian method was used. The output of agricultural goods has been proven to be significantly harmed by temperature increase. Additionally, it was seen that when the rains increased, revenues would rise. The region's total unpleseant influence of temperature is larger than its overall good spillovers of rainfall. It was discovered that a 1% increase in temperature would result in a loss of net income of Rs. 4180 every year. The relevant ramifications of the paradigm shift necessary in the agricultural sector in dry regions would be the dissemination of new farming techniques including new irrigation systems, new crop farming methods, and modified cropping patterns.

Using data gathered from the Enugu State Agricultural Development Programme (ENADP) on productivity over a forty-year period, Enete and Amusa [15] examined the effects of change of climate on the contribution of farming in Enugu State. Additionally, rainfall data from the years 1981 through 2010 were gathered to create a seasonality index and a dependability index. Utilizing descriptive statistics in conjuction with correlation analysis, the data was examined. A widespread shift of the seasonal rainfall was shown by the study.

RETRACTED

The state of rainfall pattern is defined by two main characteristics: a dependability of rainfall pattern characterized by a more pronounced fluctuation in the months of highest rainfall. These modifications are observable signs of change of climate. As rainfall continued to be increasingly unpredictable, the study once again demonstrated that except cassava and pepper, all traditional crops saw a large field drop. According to the literature study, there is a double-barrel relationship between agriculture and climate change. Farmers in Enugu will need to respond by growing new temperature-adapted species, applying insecticides, and changing the dates of planting, harvesting, and irrigation in order to lessen climate change-induced hazards to agriculture that supports national growth.

Masud [27] used samples of 500 respondents to assess the way in which the mediating influence of adaptive capacity of farmers exist between the practices of adaptation, economic, institutional limitations and technology. The study's discoveries affirmed that 67% of farmers have heard about adaptation practices but 33% are yet to hear about this development. Also, the study identified socio-economic factors and barriers such as nature, technology and institutions as the variables that hindered adaptation practices of the farmers. Akhtar et al. [28] applied PLS-SEM in analysing soico-economic and environmental interference of change of climate on the livelihoods farmers alongside their adaptive capacity in Malaysia. It was inferred from the study that the farmers had the perception of socio-economic and environmental inducements of climate change. As such, the unpleasant effects of change of climate showed an impact on farmers’ livelihoods alongside their adaptive capacity.

The study by Masud et al. [29] explored agricultural sector in Malaysia by examining how farmers perceived vulnerability to climate change alongside its spillovers on socioeconomic indices. The study used a multiple regression analysis to arrive at these submissions; the prominent indicators that have strong impacts of adaptation practices of the farmers are as follows; size of farm, age, income from farm, education level, farm experience, inadequate accessibility to extension, finances and agricultural markets. Akhtar et al. [30] investigated how farmers growing rice understand the climate change issues alongside their adaptive capacity. The authors employed a survey to conclude that farmers have moderate adaptation to climate change. Similarly, the study identified inadequate funds and insufficient information from the government were the major barriers to change of climate. This akin to the studies by Osabohie et al. [31], Imeokparia et al. [32], Osabohien et al. [33] and Matthew et al. [34].

RETRACTED

In conclusion, it is evident that studies regarding climate change and sustainable agricultural growth are very scarce within the Sahel region. Therefore, the study's hypthosis is stated as follows.

H0 there is no significant relationship between climate change and sustainable agricultural growth in the Sahel region.

H1 there is a significant relationship between climate change and sustainable agricultural growth in the Sahel region.

## 3 Methodology

### 3.1 Research design and theoretical framework

In considering the right research design for this study, an expo facto research design is used due to the kind of techanicality involved in addressing the objective of this study. Firstly, this study utilizes secondary data in which the researchers have no influence on its behavior. Similarly, the study provides information about how climate change variables explain variation in sustainable agricultural growth within the context of Sahel region.

This research work anchors on cascading climate risks theoretical framework initiated by the CASCADES research team. The framework enunciated factors that triggered climate change from the perspectives of biophysical phenomenon, meteorological variables and hydrological factors. Consequently, the framework provides a channel through which the climate change triggered factors transmit their disastrous spillovers effects on the aggregate agricultural products, livelihoods and social networks in ecosystem in one hand, and impacts transmission systems which have the tendency of escalating risks that could disperse beyond sectors and borders over the time [6].

### 3.2 Model specification

Building a model in this study to analysis the nexus between climate change and sustainable agricultural growth within a panel analysis of Sahel region requires an insight from Ricardian approach as enunciated in the works of [[31], [32], [33], [34]]. The model is specified as thus:

(1) AgriculturalOutput=f(ClimateChangeVariables)

equation (1) is adjusted to suit the purpose of this study as thus; sustainable agricultural growth replaces agricultural output, and change in rainfall, change in temperature and total emissions of greenhouse gas are used to proxy climate change variables with the inclusion of some control variables such as innovation and infrastructural development and policy variable such as government expenditure on research development, in order to improve the robustness of the model. As such, equation (1) could be re-specified as follows;

(2) SAG=f(CR,GHG,INN,IFR,GRD)

Transformation of equation (2) into a panel econometrics model results into the following equation.

(3) $${\text{SAG}}_{\text{it}}=\alpha_{0}+\beta_{1}{\text{CR}}_{\text{it}}+\beta_{2}{\text{GHG}}_{\text{it}}+\beta_{3}{\text{INV}}_{\text{it}}+\beta_{4}{\text{IFR}}_{\text{it}}+\beta_{5}{\text{GRD}}_{\text{it}}+\mu_{\text{it}}$$

in response to the pre-estimation analysis of the employed data that confirms the existence of mixture of I (0) and I (1) among the variables, this study estimated a panel autoregressive distributed lag model, following the submission of [[35], [36], [37], [38], [39]]. The ARDL model in panel form is stated as follows;

(4) $${SAG}_{it}=\sum_{i=1}^{p1}\beta_{0}{SAG}_{it-i}+\sum_{i=1}^{p1}\beta_{01}\;{LogCR}_{it-i}+\sum_{j=1}^{p2}\beta_{02}{LogGHG}_{it}+\sum_{k=1}^{p3}\beta_{03}\;{INV}_{it}+\sum_{k=1}^{p3}\beta_{04}\;{IFR}_{it}+\sum_{i=1}^{p1}\beta_{05}\;{GRD}_{it}+\theta {ECM}_{it}+\sum_{i=1}^{p1}\beta_{6}\Delta {SAG}_{it-i}+\sum_{j=1}^{p2}\beta_{7}{\Delta \mathrm{Log}\;CR}_{it}+\sum_{k=1}^{p3}\beta_{8}\Delta {logGHG}_{it}+\sum_{i=1}^{p1}\beta_{9}\Delta {LogINV}_{it}+\sum_{j=1}^{p2}\beta_{10}\Delta \mathrm{Log}\;{IFR}_{it}+\sum_{k=1}^{p3}\beta_{11}\Delta \mathrm{Log}\;{GRD}_{it}+u_{t}$$

Note β_0_ to β_05_ represents the long run parameters, β_6_ to β_11_ represents the short run parameters and θ represents coffecient of the speed of adjustment which is expected to be negative and significant.

RETRACTED

### 3.3 Causality between climate change and sustainable agricultural growth

In establishing the direction of climate change variables and sustainable agricultural growth in Sahel region, the key variables of interest in this study were subjected to panel Granger causality, in which their models were specified into model 4–6 as follows;

(5) $${\text{SAG}}_{\text{it}}=\alpha_{0}+\sum_{i=1}^{n}\alpha_{i}{\text{SAG}}_{2\text{it}-i}+\sum_{j=1}^{n}\beta_{j}{\text{CR}}_{\text{it}-j}+\sum_{k=1}^{n}\delta_{k}{\text{GHG}}_{\text{it}-k}+U_{1\text{it}}$$

(6) $${\text{CR}}_{\text{it}}=\alpha_{0}+\sum_{i=1}^{n}\alpha_{i}{\text{CR}}_{2\text{it}-i}+\sum_{j=1}^{n}\beta_{j}{\text{SAG}}_{\text{it}-j}+\sum_{k=1}^{n}\delta_{k}{\text{GHG}}_{\text{it}-k}+U_{2\text{it}}$$

(7) $${\text{GHG}}_{\text{it}}=\alpha_{0}+\sum_{i=1}^{n}\alpha_{i}{\text{GHG}}_{2\text{it}-i}+\sum_{j=1}^{n}\beta_{j}{\text{CR}}_{\text{it}-j}+\sum_{k=1}^{n}\delta_{k}{\text{SAG}}_{\text{it}-k}+U_{1\text{it}}$$

Moreover, it is important to state the apriori expections of the study in order to see if the empirical investigation within sahel region is in tandem or otherwise with the aprori expectaions. This is summarised as follows in Table 1 below.

RETRACTED

**Table 1:** A priori expectations and Data Source.

Abbreviation	Variables	Parameters	Expected Value
CR	Change in Rainfall	$\beta_{1}$	Positive (+)
GHG	Greenhouse Gas	$\beta_{2}$	Negative (−)
INV	Innovation	$\beta_{3}$	Positive (+)
IFR	Infrastructural Development	$\beta_{4}$	Positive (+)
GRD	Government Expenditure on R&D	$\beta_{5}$	Positive (+)

In providing detailed information about how the variables of the study are defined operatonally, efforts have been made to summarize how these variables have been proxied in Table 2 below.

**Table 2:** Measurement and operation definitions of variables.

**Abbreviation**	**Description of Variables**
SAG	Sustainable Agricultural Growth. This is proxied by agriculture, forestry, and fishing value added as a percentage of GDP. Its unit of measurement is percentag
CR	Change in Rainfall. This is measured by average precipitation in depth in MM per year
GHG	Greenhouse Gas. This is measured by total greenhouse gas emission
INV	Innovation. The number of individuals who have access to internet as percentage of total population is used to proxy it, as percentage is its measurement
IFR	Infrastructural Development. The number of individual who have access to electricity as percentage of total population. Percentage is the unit of its measurement
GRD	Government Expenditures on Research and Development. This is measured by the government's capital and recurrent spending on education as percentage of government expenditure. Its unit is in percentage.

### 3.4 Source of data and scope of the study

In investigating the relationship between climate change and sustainable agricultural growth in Sahel region using secondary data, this study used annual time series data within the periods of 1990 and 2020. All the data were collected from World Development Indicators (WDI). Consquenntly, data from 9 countries out of 13 countries within Sahel region were collated. It is needful to stress that the inclusion of these countries in the study was based on data available on the variables of interest. The countries selected are: Burkina Faso, Chad, Eritrea, Mali, Mauritania, Niger, Nigeria, Senegal and Sudan. The observed missing data of some variables were addressed by following the technique of Benchani and Swiss (2019) in filling missing data in panel study. To this end, the study employs the average of the last four most recent years in the dataset to replace the missing points. This technique makes the panel dataset to be strongly balanced, and eventually contributes to the possibility of the balanced panel analysis in this study.

RETRACTED

## 4 Results and discussion

This section provides detailed analysis and discussion of the results, alongside the policy recommendation of the study.

Table 3 shows the description of various statistics associated with the dataset in the study, so we can determine whether the dataset is in agreement to the assumption of the normal distribution. Steaming from the above results, the following variables the annual change in rainfall in log form, greenhouse gas in log form, government expenditure on research and development, sustainable agricultural growth and infrastructural development are moderately dispersed from their mean. This is because the values of the standard deviation of these set of the variables are less than the values of their mean. Whereas, innovation data dispersed widely from the mean, because its mean value is less than the standard deviation.

**Table 3:** Descriptive statistics.

Descriptive Statistics	LCR	LGHG	INV	GRD	SAG	IFR
Mean	5.853	10.186	4.673	3.304	28.235	25.328
Median	5.774	10.034	0.522	2.600	27.241	22.886
Maximum	7.050	12.668	42.600	10.300	55.771	70.400
Minimum	4.477	8.2133	1.320	1.000	10.642	1.100
Std. Deviation	0.767	1.1057	8.716	1.943	10.092	17.419
Skewness	−0.151	0.5954	2.383	1.513	0.405	0.470
Kurtosis	2.103	2.8150	8.264	4.939	2.567	2.129
Jargue-Bera	10.06	16.338	567.388	145.446	9.503	18.468
Probability	0.006	0.0002	0.000	0.000	0.008	0.000
Sum	1580.491	2750.370	1261.798	892.286	7623.632	6838.687
Sum Sq. Dev.	158.634	328.893	20439.65	1016.153	27401.50	81620.38
Observations	279	279	279	279	279	279

In the same vein, except the annual change in rainfall, all other variables are skewed in a positive direction. The values of kurtosis of various dataset show that the annual change in rainfall, greenhouse gas, sustainable agricultural growth and infrastructural development are platykurtic in their distribution. However, those of government expenditures on research and development and innovation possess leptpkurtic distributions. In conclusion, the majority of the dataset shows some level of agreement with the assumption of normal distribution.

Table 4 presents the outcomes of the correlation analysis of the various pairs of explanatory variables used in this study. From the table above, it could be reported that the degrees of correlation that exists between different pairs of the regressors are so low that the highest correlation in the table is 0.652. This implies that the subsequent regression will be freed from the problem of multicollinearity as reinforced by the submission of [38] claiming that it is only the pair of regressors with correlation of 0.9 has capacity cause multcollienarity in a model.

RETRACTED

**Table 4:** Correlation matrix among independent variables.

	LCR	LGHG	IFR	INV	GRD
LCR	1.000	0.442	0.368	0.137	0.652
LGHG	0.442	1.000	0.274	0.284	0.587
IFR	0.368	0.274	1.000	0.579	0.554
INV	0.137	0.284	0.579	1.000	0.322
GRD	0.652	0.587	0.554	0.322	1.000

It has been observed over the time that one of the serious dangers non-staionary time series data poised to empirical analysis is spurious or nonsense regression. This problem diminishes the validity of empirical work in terms of its relevance and policy implication. This paper aims to overcome this problem by subjecting the stationarity properties of the study's data to the pre-estimation check using relevant panel unit root tests- Levin, Lin & Chu t* Test and Im, Pesaran and Shin W-stat tests respectively. According to the estimated results in Table 5, the following set of variables, GRD, LCR and SAG are free from unit root. On the other hand, LGHG, IFR and INV possess unit root. This confirms that the variables have mixed stationary properties of I(0) and I(1), which could cause the variables to exhibit a divergence in the short run.

**Table 5:** Panel unit root tests.

Variable	Level	Prob.	1st Diff.	Prob.	Remark
LGHG	5.342	1.000	−16.716	0.000	I(1)
GRD	−2.483	0.006	–	–	I(0)
LCR	−9.840	0.000	–	–	I(0)
IFR	1.576	0.942	0.736	0.769	I(1)
INV	5.551	1.000	−0.643	0.259	I(1)
SAG	−3.370	0.000	–	–	I(0)
**Im, Pesaran and Shin W-stat Test**					
LGHG	−0.344	0.365	−19.523	0.000	I(1)
GRD	−19.523	0.000	–	–	I(0)
LCR	−15.280	0.000	–	–	I(0)
IFR	−0.097	0.461	−11.085	0.000	I(1)
INV	1.741	0.959	−6.401	0.000	I(1)
SAG	−2.584	0.004	–	–	I(0)

Having established the possibility of the short run divergence due to unit root problem among some varibales in the previous table, further effort was made to test for the possibility of a long run convergence among these variabls using Johansen Fisher Panel Cointegration test. As reported in Table 6, it could be inferred that the presence of at most 5 cointegrating equations existed in the estimated model. This result reinforces the existence of convergence among the variables of interest in thelong run.

**Table 6:** Johansen Fisher panel cointegration test.

Hypothesized No. Of CE(s)	Trace test	Prob.	Max-eigen test	Prob.
None	250.1	0.000	111.4	0.000
At most 1	133.5	0.000	76.75	0.000
At most 2	72.62	0.000	39.71	0.002
At most 3	44.58	0.000	34.19	0.011
At most 4	24.46	0.140	20.57	0.301
At most 5	24.64	0.135	24.64	0.135

The estimation of a panel ARDL requires the use of the appropriate and optimal number of lags so as not to undermine the achievement of the best results. Against the backdrop, this study utilized the Akaike Information Criteria to determine the appropriate and optimal number of lags for the ARDL estimation. As indicated in Fig. 1, the lag one (1) was considered as the appropriate and optimal lag that could guarantee the best estimation.

RETRACTED

**Fig. 1:** Var lag order selection criteria.

Source: Authors’ (2022)

The estimation of a panel ARDL of the relationship between climate change and sustainable agricultural growth within Sahel region was reported in Table 7. Firstly, greenhouse gas followed the aprori expectation in the short run, while showing otherwise in the long run. Change in rainfall did not follow the aprori expectation in the both short run and the long run. Also, the speed of adjustment between the short run and the long run had appropriate sign and significant as well. This means that 27% of the short run disequilibrium in the relationship between climate change and sustainable agricultural growth due to error, was adjusted in the long run. Furthermore, greenhouse gas emission had an insignificant negative relationship with sustainable agricultural growth in the short run.

**Table 7:** Panel ARDL estimation of climate change and sustainable agricultural growth in sahel region.

Regressors	Long Run Coefficient	T-statistics	Prob.	Short Run Coefficient	T-statistics	Prob.
LGHG	7.690*	4.277	0.000	−3.422	0.824	0.410
INV	−0.033	0.285	0.775	−0.277	0.624	0.533
LCR	−22.032*	6.874	0.000	−20.427***	1.871	0.062
GRD	0.160	0.283	0.776	−0.895***	1.784	0.076
IFR	−0.219*	3.371	0.000	0.050	0.433	0.664
ECM(-1)	−0.277**	3.122	0.002			

Notes: *Significant at1% **significant at 5% ***Significant at 10%.

Meanwhile, in the long run, the relationship became positive and significant. However, change in rainfall had both short run and long run negative relationship with sustainable agricultural growth. Innovation had insignificant negative relationship with sustainable agricultural growth in both the short run and the long run. Government expenditure on research and development had negative relationship with sustainable agricultural growth, which is significant at 10% level of significance in the short run, but showed otherwise in the long run. Infrastructural development had an insignificant positive relationship with sustainable agricultural growth in the short run, but this relationship became negative and significant in the long run.

Therefore, this study submits that climate change orchestrated by change in rainfall is a very strong factor causing reduction in sustainable agricultural growth in the Sahel region. Whereas, greenhouse gas is not a serious factor affecting sustainable agricultural growth in the Sahel region. By and large, climate change is a militating factor against sustainable agricultural growth in Sahel region. This conclusion is supported by similar past empirical works such as Alboghdady and El-Hendawy [24] focusing on the Middle East and North Africa, Chandio et al. [12] which focused on China, Belloumi [14] focused on 11 Eastern and Southern Africa and Ayinde et al. [19], Yu and Osabohien [40], Matthew et al. [41], Edafe et al. [42], Osaboohein [43], Osabohien [44] and Ju et al. [45], focused on Nigeria and Africa. Despite the fact that different methodology was utilized in this study. However, the findings in this study are contrary to the submission of the following Zhai and Zhuang [18] and Molua [16] in related studies in South East Asia and Africa respectively.

RETRACTED

In checking the robustness of the results obtained from the panel ARDL long run estimations, Panel DOLS was carried out while employing the same dataset, the results of which are presented in Table 8. The coefficient of LGHG was positive and significant in the result of panel DOLS model as in the result of the panel ARDL. Similarly, the coefficients of LCR, INV and IFR were positive in the Panel DOLS results. This also reinforces the valitidity of the results of the panel ARDL.

**Table 8:** Robustness check (results of panel dynamic least squares (DOLS)).

Regressors	Coefficient	T-Statistics	Prob.
LGHG	9.927**	2.979	0.003
GRD	−2.597**	2.339	0.021
LCR	−8.199	0.643	0.521
INV	−0.009	0.035	0.971
IFR	−0.159	1.522	0.131
R- squared	0.917		

Notes: *Significant at1% **significant at 5% ***Significant at 10%.

In this section, further effort was made to determine the flow of information among the climate change variables and sustainable agricultural growth in Sahel region via the technique of Pairwise Dumitrescu Hurlin Panel Causality Tests. The findings in Table 9 enunciated that unidirectional causal relationship flows from sustainable agricultural growth to change in rainfall. In the same vein, one way feedback relationship flows from sustainable agricultural growth to greenhouse gas emission. Meanwhile, change in rainfall unidirectionally Granger causes greenhouse gas emission. From the above scenario, inference could be drawn from the study that the emergence of climate change in Sahel region could be orchestrated in the future as a result of agricultural activities which involve ecological disturbance via deforestation, fishing etc.

**Table 9:** Pairwise dumitrescu hurlin panel causality tests of climate change variables and sustainable agricultural growth in sahel region.

Null hypothesis	W-Stat	Prob.	Decision	Causality
LCR →SAG	7.976	0.613	H0 Accepted	
SAG →LCR	0.622	0.041	H0 Rejected	Unidirectional
LGHG →SAG	7.875	1.E−12	H0 Accepted	
SAG→ LGHG	11.281	0.000	H0 Rejected	Unidirectional
LGHG →LCR	1.429	0.343	H0 Accepted	
LCR →LGHG	25.704	0.000	H0 Rejected	Unidirectional

Note: **→** means does not homogeneously cause.

RETRACTED

## 5 Summary, conclusion and policy implications

In providing an empirical answer to the question of whether nexus exists between climate change and sustainable agricultural growth in Sahel region between 1990 and 2020, this study utilized suitable econometrics techniques – Panel ARDL and Pairwise Dumitrescu Hurlin Panel Causality Tests to address the objective of this study with following conclusions; firstly, the climate change orchestrated by change in rainfall is a very strong factor causing reduction in sustainable agricultural growth in the Sahel region. Whereas, greenhouse gas emission is not a prominent factor causing a negative impact on sustainable agricultural growth in the Sahel region. In addition, a unidirectional causal relationship flows from sustainable agricultural growth to change in rainfall. In the same vein, one way feedback relationship flows from sustainable agricultural growth to greenhouse gas emission. Meanwhile, change in rainfall unidirectionally Granger causes greenhouse gas emission. Therefore, agricultural activities which involve ecological disturbance-deforestation and indiscriminate fishing have the capacity to bring the emergence of climate change in Sahel region in the nearest future.

In the light of the above findings, this study recommends that, in addressing the adverse effects of change in rainfall on agricultural sustainability, the policymakers in Sahel region in particular and Africa as a whole should embark on a policy mix by embanking on mitigating policy response towards ensuring sustainable agricultural production via irrigation which is the best mode of water provisions without causing negative spilliovers on the environment. Also, since agriculture is the principal source of livelihood of the Sahel residents, the policymakers should be proactive by embarking on policies and programs that would build the resilience and adaptation of the region ahead of the future adverse effects of agriculturally induced climatic change. The limitation of this study is in its scope of coverage. However, future studies could be extended further to other newly emerging and industrialized economies.

## Informed consent

Not applicable.

## Ethical approval

Not required.

## Author contribution statement

Ting Wang, Chengwu Sun, Zheqi Yang: Conceived and designed the analysis; Analyzed and interpreted the data; Contributed analysis tools or data; Wrote the paper.

RETRACTED

## Data availability statement

Data will be made available on request.

## Additional information

No additional information is available for this paper.

## Declaration of competing interest

The authors declare no conflcit of interest.

## References

[1] Intergovernmental Panel on Climate Change (IPCC) (2007). http://www.ipcc.ch.

[2] Carter C., Cui X., Ghanem D., Mérel P. (October 2018). Identifying the economic impacts of climate change on agriculture. Annual Review of Resource Economics.

[3] Pachauri R.K., Allen M.R., Barros V.R., Broome J., Cramer W., Christ R., Church J.A., Clarke L., Dahe Q., Dasgupta P. (2014). Climate change 2014: synthesis report. Contribution of Working Groups I, II and III to the ﬁfth assessment report of the IntergovernmentalPanelonClimateChange. IPCC.

[4] Sartori N., Fattibene D. (2019).

[5] USAID (2017). Climate change risk profile. West Africa Sahel (Regional fact sheet).

[6] Hidden M., Lahn G., Carter T.R., Klein R.J.T., Otto I.M., Pohl B., Reyer C.P., Tondel O., Cascading F. (2020).

[7] Pye O. (2020). https://www.cer.eu/sites/default/files/pbrief_sahel_31.3.21.pdf.

[8] Ayinde O.E., O O., Ajewole I., Ogunlade M. O. Adewumi (2010). Empirical analysis of agricultural production and climate change: a case study of Nigeria. J. Sustain. Dev. Afr..

[9] Busby J. (2018). Taking stock: the field of climate and security. Curr. Clim. Change Rep..

[10] Biasutti M. (2019).

[11] Cooper R., Price R.A. (2019). http://opendocs.ids.ac.uk/opendocs/handle/123456789/14585.

[12] A A., Chandio Y., Jiang A., Rehman A. Rauf (2020). Short and long-run impacts of climate change on agriculture: an empirical evidence from China. International Journal of Climate Change Strategies and Management.

[13] Agbola P., Fayiga A.O. (2016). Effects of climate change on agricultural production and rural livelihood in Nigeria. Journal of Agricultural Research and Development.

[14] Belloumi M. (2014).

[15] Enete A.A., Amusa T.A. (2010). Challenges of agricultural adaptation to climate change in Nigeria: a synthesis from the literature. Field Actions Science Reports. The Journal of Field Actions.

[16] Molua E.L., Benhin J.K., Kabubo-Mariara J., Ouedraogo M., El-Marsafawy S. (2010). Global climate change and vulnerability of African agriculture: implications for resilience and sustained productive capacity. Q. J. Int. Agric..

[17] Apata T.G. (2011). Effects of global climate change on Nigerian agriculture: an empirical analysis. CBN Journal of Applied Statistics.

[18] Zhai F., Zhuang J. (2012). Agricultural impact of climate change: a general equilibrium analysis with special reference to Southeast Asia. Climate change in Asia and the Pacific: How can countries adapt.

RETRACTED

[19] Ayinde O.E., Muchie M., Olatunji G.B. (2011). Effect of climate change onagricultural productivity in Nigeria: a co-integration model approach. J. Hum. Ecol..

[20] Atedhor G.O. (2015). Agricultural vulnerability to climate change in Sokoto State, Nigeria. Afr. J. Food Nutr. Sci..

[21] Onyeneke R.U., Nwajiuba C.A., Emenekwe C.C., Nwajiuba A., Onyeneke C.J., Ohalete P., Uwazie U.I. (2019). Climate change adaptation in Nigerian agricultural sector: a systematic review and resilience check of adaptation measures. AIMS Agriculture and Food.

[22] Ozor N., Madukwe M.C., Enete A.A., Amaechina E.C., Onokala P., Eboh E.C., Garforth C. (2012). A framework for agricultural adaptation to climate change in Southern Nigeria. Int. J. Agric. Sci..

[23] Belloumi M. (2014). Investigating the linkage between climate variables and food security in ESA countries. Reg. Environ. Change.

[24] Alboghdady M., El-Hendawy S.E. (2016). Economic impacts of climate change and variability on agricultural production in the Middle East and North Africa region. International Journal of Climate Change Strategies and Management.

[25] Pickson R.B., Boateng E. (2022). Climate change: a friend or foe to food security in Africa?. Environ. Dev. Sustain..

[26] Shakoor U., Saboor A., Ali I., Mohsin A.Q. (2011). Impact of climate change on agriculture: empirical evidence from arid region. Pakistan J. Agric. Sci..

[27] Masud M.M., Akhtar R., Al Mamun A., Uddin M., Siyu L., Yang Q. (2022). Modelling the sustainable agriculture management adaptation practices: using adaptive capacity as a mediator. Front. Environ. Sci..

[28] Akhtar R., Masud M.M., Rahman M.K. (2022). Farmers' livelihood and adaptive capacity in the face of climate vulnerability. Journal of Social Economics.

[29] Masud M.M., N Azam M., Mohiuddin M., Banna H., Akhtar R., Alam A.F., Begum H. (2017). Adaptation barriers and strategies towards climate change: challenges in the agricultural sector. J. Clean. Prod..

[30] Akhtar R., Masud M.M., Afroz R. (2019). Perception of climate change and the adaptation strategies and capacities of the rice farmers in Kedah, Malaysia. Environment and Urbanization ASIA.

[31] Osabohien R., Matthew O., Aderounmu B., Olawande T. (2019). Greenhouse gas emissions and crop production in West Africa: examining the mitigating potential of social protection. Int. J. Energy Econ. Pol..

[32] Imeokparia L., Olaoye O.P., Bello B.A., Osabohien R., Aderemi T.A., Gershon O., Abidemi A. (2023). A panel analysis of crude oil exports and poverty reduction in african oil producing countries: implication for the sustainable development goal one. Int. J. Energy Econ. Pol..

RETRACTED

[33] Osabohien R., Karakara A.A.W., Ashraf J., Al-Faryan M.A.S. (2023). Green environment-social protection interaction and food security in Africa. Environ. Manag..

[34] Aderemi T.A., Alejo A., Omoyele O.S., Olaoye O.P., Olanipekun W.D., Azuh D.E. (2022). An econometric analysis of clean energy supply and industrial development in Nigeria: implications for sustainable development. Int. J. Energy Econ. Pol..

[35] Pesaran M.H., Shin Y., Smith R.J. (2001). Bounds testing approaches to the analysis of level relationships. J. Appl. Econom..

[36] Pesaran M., Pesaran B. (1997).

[37] Pesaran H., Shin Y., Smith R. (1999). Pooled Mean Group estimation anddynamic heterogeneous panels. Journal of the American Statistical Asssociation.

[38] Qingyan Y., Anser M.K., Abbas S., Ashraf J., Ahmad M., Jamshid J., Osabohien R. (2022). Integrating the role of green fiscal policies with energy prices volatility and energy efficiency: presenting a COVID-19 perspective. Front. Energy Res..

[39] Osabohien R., Matthew O., Adegboye F., Odularu G. (2020). Agricultural value added, food and nutrition security in west Africa. Realizing the SDG 2. Nutrition, Sustainable Agriculture and Climate Change in Africa: Issues and Innovative Strategies.

[40] Yu Z., Osabohien R. (2023). Investigating the impact of education and women in agriculture on human capital outcomes in Africa: an interaction analysis. Problemy Ekorozwoju/Problems of Sustainable Development.

[41] Matthew O., Osabohien R., Omosehin O.O., Jawaid N., Aderemi T., Olanrewaju O., Evans-Osabuohien P.N. (2023). Information and communication technology deployment and agricultural value chain nexus in Nigeria. Heliyon.

[42] Edafe O.D., Osabuohien E., Matthew O., Osabohien R., Khatoon R. (2023). Large-scale agricultural investment and female employment in African communities: quantitative and qualitative insights from Nigeria. Land Use Pol..

[43] Osabohien R. (2023). ICT adoption and youth employment in Nigeria's agricultural sector. African J. Econ. Manag. Stud..

[44] Osabohien R. (2022). Soil technology and post-harvest losses in Nigeria. J. Agribus. Dev. Emerg. Econ..

[45] Ju P., K Anser M., Osabohien R., Ochuba O., R Ahuru R., Ashraf J. (2022). Trade openness, foreign direct investment and sustainable agriculture in Africa. Problemy Ekorozwoju.

